The article "MiRNA-211 suppresses cell proliferation, migration and invasion by targeting SPARC in human hepatocellular carcinoma" was retracted in 2023. Reasons: duplicated images; duplicated data; original data or images not available.

# MiRNA-211 suppresses cell proliferation, migration and invasion by targeting SPARC in human hepatocellular carcinoma

**DOI:** 10.1038/srep26679

**Published:** 2016-05-27

**Authors:** Biao Deng, Lei Qu, Jinfang Li, Jiaqing Fang, Shouwen Yang, Zhongwei Cao, Zhechuan Mei, Xing Sun

**Affiliations:** 1 Department of General Surgery, Shanghai First People’s Hospital, Shanghai Jiao Tong University, 100 Haining Road, Shanghai, 200080, China; 2 Department of Neurology, The Second Affiliated Hospital, Chongqing Medical University, Chongqing, China; 3 Department of Gastroenterology, Tianyou Hospital, TongJi University, 500 Zhennan Road, Shanghai, 200331, China; 4 Department of Gastroenterology, Shanghai First People’s Hospital, Shanghai Jiao Tong University, 100 Haining Road, Shanghai, 200080, China; 5 Department of Gastroenterology, The Second Affiliated Hospital, Chongqing Medical University, Chongqing, China

## Abstract

Previous studies have shown that the expression of miR-211 was downregulated in hepatocellular carcinoma (HCC). However, the molecular function and mechanism of miR-211 in HCC growth and invasion are largely unclear. We found that miR-211 is downregulated in HCC tissues and cell lines, respectively. Further results showed that low miR-211 associated with TNM stage, vein invasion status, and poor prognosis. Ectopic expression of miR-211 effectively suppressed HCC cell proliferation, migration and invasion both *in vitro* and *in vivo*. We identified SPARC as a bona fide target of miR-211, and overexpression of miR-211 decreased the mRNA and protein expression of SPARC. Finally, we confirmed that the overexpression of SPARC in miR-211-expressing HCC cells can partially restore the inhibitory effect of miR-211. Taken together, our results demonstrated that loss of miR-211 expression and thus uncontrolled SPARC overexpression might drive progression of HCC, which may provide a novel therapeutic strategy for the treatment of HCC.

Hepatocellular carcinoma (HCC) is one of the common malignant primary liver tumors and the third leading cause of death from cancer worldwide, particularly in East Asia and South Africa^1^. It has been demonstrated that tumorigenesis was caused by amplification of oncogenes and/or loss of tumor suppressors, however, the molecular and cellular mechanisms remain largely unknown^2^,^3^,^4^. Despite significant improvement in the survival rates of patients with HCC, metastasis or recurrence is frequently observed^1^. Understanding the mechanisms of crucial genes is necessary for further elucidating the pathogenesis of HCC and may offer an opportunity to develop novel therapeutic strategies.

MicroRNAs are highly conserved, endogenous small non-coding RNAs that negatively regulate gene expression at the posttranscriptional level and thereby participate in the control of various biological processes, such as cell growth, cell motility, apoptosis, and stress response^5^,^6^,^7^. Many studies have shown that deregulation of miRNAs occurs in a wide range of human diseases, including carcinogenesis, and that altered miRNA expression plays important roles in HCC progression and directly regulated cell growth and metastasis^7^,^8^,^9^,^10^,^11^,^12^. The roles of miR-211 in tumor progression can be considered quite contradictory. Previous reports have demonstrated that the expression level of miR-211 was significantly decreased in many tumors, such as glioma, melanoma, ovarian cancer and hepatocellular carcinoma^13^,^14^,^15^,^16^. However, miR-211 was upregulated in head and neck squamous cell carcinoma (HNSCC) and directly regulated TGFβRII to promote HNSCC progression and enhance c-Myc expression^17^. Recent studies have demonstrated that overexpression of miR-211 promoted colorectal cancer cell growth by downregulating the expression level of the CHD5 tumor suppressor *in vitro* and *in vivo*. However, the expression of miR-211 in colorectal cancer tissues was not clear^18^. The effect and underlying molecular mechanisms of miR-211 in regulating hepatocellular carcinoma development are poorly understood.

The article "MiRNA-211 suppresses cell proliferation, migration and invasion by targeting SPARC in human hepatocellular carcinoma" was retracted in 2023. Reasons: duplicated images; duplicated data; original data or images not available.

Secreted protein acidic and rich in cysteine (SPARC) belongs to the matricellular family of secreted proteins that regulates cell adhesion, migration, tissue repair and remodeling^19^. SPARC is considered as an oncogene because it is highly expressed in various tumors including glioma, prostate, and gastric carcinomas^20^,^21^,^22^. Meanwhile, high SPARC is also found to be associated with aggressive stages of melanoma and is correlated with poor prognosis^23^. Similarly, a recent study has pointed that neoplastic-produced SPARC boosted the invasive and metastatic potentials of a cancer stem cell-enriched subpopulation in prostate cancer cells^24^. It has been reported that SPARC repressed E-Cadherin leading to a migratory and invasive behavior^25^. SPARC is reported to be upregulated in HCC both at mRNA and protein levels^26^,^27^. However, previous study has shown that SPARC overexpression inhibited HCC cellular aggressive features and enhanced HCC cells sensitivity to 5-FU-based chemotherapy^28^. Therefore, it would be interesting to investigate the regulatory mechanism of SPARC in HCC.

In this study, we indicated that miR-211 is a tumor suppressor that is pathologically down-regulated in HCC and cell lines. Ectopic expression of miR-211 inhibits HCC cell proliferation and invasion capability *in vitro* and *in vivo*. Furthermore, we show that SPARC is a direct target of miR-211. Therefore, our results suggest that miR-211 might play important functions in HCC progression and represent a potential target for HCC therapy.

The article "MiRNA-211 suppresses cell proliferation, migration and invasion by targeting SPARC in human hepatocellular carcinoma" was retracted in 2023. Reasons: duplicated images; duplicated data; original data or images not available.

## Results

### MiR-211 is downregulated in primary HCC cell lines and tissues

The expression levels of miR-211 were first determined by real-time quantitative PCR in five hepatocellular cell lines. As shown in Fig. 1A, the expression of miR-211 was strongly downregulated in the all HCC cell lines compared with the normal hepatic cell line LO2, especially in the highly metastatic HCC cell lines, MHCC-97H and MHCC-LM3. In order to further explore that miR-211 expression levels differ between tumor and non-tumor tissues, we examined the expression in 227 pairs of HCC tissues and adjacent non-neoplastic liver tissues. Consistently, the results showed that miR-211 is significantly downregulated (P < 0.001) in HCC tissues compared with that in the paired adjacent non-tumorous tissues (Fig. 1B). These results indicate that miR-211 showed reduced expression levels in HCC.

### MiR-211 downregulation is associated with HCC clinicopathological features and poor overall survival of HCC patients

To assess whether miR-211 has any prognostic significance, we analyzed the correlation between miR-211 levels and the clinicopathologic features of HCC patients. As shown in Table 1, miR-211 expression was significantly associated with vein invasion (P = 0.0028) and TNM stage (P = 0.0004). Patients with high miR-211 expression displayed significantly higher overall survival (OS) (median survival time of 64.0 months) probability than those with low miR-211 expression (median survival time of 45.0 months, P < 0.0001) (Fig. 1C) based on Kaplan-Meier analysis. Moreover, HCC patients with low miR-211 expression exhibited notably shorter overall survival than those with high expression of miR-211 in either the stage I-II subgroup (n = 138; P < 0.0001) (Fig. 1D) or the stage III-IV subgroup (n = 89; P = 0.0006) (Fig. 1E). These results indicated that miR-211 might contribute to HCC progression and metastasis.

### MiR-211 inhibits tumor cell growth *in vitro* and *in vivo*

To further understand the functional significance of miR-211 in HCC, we established stable cells to restore the expression of miR-211 in both MHCC-LM3 (LM3) and MHCC-97H (97H) cells, which had low endogenous miR-211 expression, and the overexpression levels of miR-211 were confirmed by real-time quantitative PCR (Fig. 2A). We then investigated the effect of miR-211 on HCC cell proliferation. Ectopic miR-211 expression significantly suppressed cell proliferation compared with cells expressing control vector in 97H and LM3 cells (Fig. 2B). To assess the long-term effect of miR-211 on cell growth, the colony formation assay revealed that miR-211 overexpression dramatically attenuated growth abilities of the HCC cells, based on the number and the size of the measured formed colonies (Fig. 2C). In addition, miR-211 overexpression induced an increase of apoptotic cells in 97H and LM3 cells (Fig. 2D). Moreover, the role of miR-211 in tumor growth was determined *in vivo*. The stable cells either overexpressing LM3-miR-211 or expressing the control vector LM3-vector were injected subcutaneously into the flank of nude mice. Our data indicated that miR-211 dramatically inhibited tumor growth, as evidenced by the sizes and weights of dissected tumors (Fig. 2E). In addition, immunostaining demonstrated that the tissues from the miR-211 group showed weaker Ki-67 expression than that in tissues from the vector group (Fig. 2F). These data strongly supported the hypothesis that miR-211 acted as a tumor suppressor that can suppress tumor growth *in vitro* and *in vivo*.

The article "MiRNA-211 suppresses cell proliferation, migration and invasion by targeting SPARC in human hepatocellular carcinoma" was retracted in 2023. Reasons: duplicated images; duplicated data; original data or images not available.

### Overexpression of miR-211 suppresses HCC cell migration and invasion *in vitro* and *in vivo*

To define the biological effect of miR-211 downregulation on metastasis in HCC patients, wound healing and transwell assay were performed. Consistent with clinical features, miR-211 overexpression drastically decreased the migration speed in the two tested cell lines (by ∼50% in the 97H cell line and by ∼45% in the LM3 cell line) at 24 h compared with the vehicle control (Fig. 3A). The Matrigel-coated transwell assay also confirmed that miR-211 overexpression markedly inhibited the invasive capacity of the 97H and LM3 cancer cell lines (Fig. 3B). To further determine the effect of miR-211 on the metastatic properties *in vivo*, we chose the HCC cell line LM3, which has the propensity to form lung metastases and is used as a model of HCC metastasis. The LM3-miR-211 cells, as well as their corresponding vector control cells, were injected into nude mice via tail vein. Strikingly, histological staining of lung tissue with H&E showed that mice injected with LM3-miR-211 cells displayed no visible metastasis in their lungs, whereas large hepatic tumors were found in mice injected with control LM3-vector cells (Fig. 3C). Taken together, both the *in vitro* and *in vivo* studies implied that miR-211 plays a suppressive role in HCC metastasis.

### SPARC is direct target of miR-211

To investigate the molecular mechanisms by which miR-211 may regulate HCC growth and metastasis, systemic bioinformatic algorithms (TargetScan, miRDB) were applied to analyze and identify potential targets. For further analysis, we chose SPARC, which contain putative miR-211 complementary sites and play an important role in cancer progression (Fig. 4A). To validate whether SPARC is a bona fide targets of miR-211 in HCC, we tested the luciferase activities of SPARC using a dual-luciferase reporter assay. As expected, miR-211 remarkably reduced the luciferase activities of wild-type 3′UTR of SPARC, whereas this effect was largely eliminated when the binding sites in SPARC 3′-UTR targeted by miR-211 were mutated (Fig. 4B). Conversely, after cotransfection with the miR-211 inhibitor with the reporter plasmid in 97H-miR-211 cells, the relative luciferase activity of the reporter containing wild-type SPARC 3′-UTR was obviously increased while the luciferase activity of the mutant SPARC had no significant change (Fig. 4C). Consistent with these results, a decrease of endogenous SPARC mRNA was observed by real-time quantitative PCR (Fig. 4D). We also found that forced expression of miR-211 dramatically decreased the endogenous protein levels of SPARC in 97H and LM3 cells (Fig. 4E). Moreover, the inhibition of miR-211 in 97H-miR-211 and LM3-miR-211 cells by transfecting the miR-211 inhibitor increased SPARC protein expression (Fig. 4F). These results indicated that miR-211 directly targets SPARC and represses its expression.

The article "MiRNA-211 suppresses cell proliferation, migration and invasion by targeting SPARC in human hepatocellular carcinoma" was retracted in 2023. Reasons: duplicated images; duplicated data; original data or images not available.

### SAPRC acts as an oncogene in HCC cells and is inversely correlated with the expression of miR-211 in HCC tissues

Next we sought to investigate the expression levels of SPARC in the same panel of 227 pairs of HCC tissue samples. The expression levels of SPARC mRNA were significantly higher in human HCC samples than in the paired adjacent non-tumor tissue samples (Fig. 5A). Furthermore, a statistically significant inverse correlation was revealed between mRNA levels of SPARC and miR-211 by Spearman’s correlation analysis (Fig. 5B). To further validate this finding, we performed IHC analysis to detect the protein expression of SPARC in consecutive tissue microarray slides consisting of the 227 HCC samples (Fig. 5C). Consistent with previous results, the statistical analysis also revealed that the expression of SPARC protein was significantly inversely correlated with miR-211 levels in the HCC samples (Fig. 5D). The results indicated that the loss of miR-211 that resulted in SPARC over-expression may be critical to HCC development. To investigate the functional significance of SPARC in the proliferative and invasive capability of HCC cell lines induced by miR-211, we performed RNA interference based silencing of both SPARC in 97H and LM3 cells and confirmed the expression of SPARC by western blot (Fig. 5E). As expected, apoptosis analysis using flow cytometry assay showed SPARC silencing led to an increased percentage of apoptotic cells (Fig. 5F). We also found that siRNA mediated knockdown of SPARC resulted in a significant reduction in cell migration and invasion ability compared to 97H and LM3 cells transfected with negative control (SCR) (Fig. 6G,H). These results suggest that SPARC were all upregulated in HCC and might function as an oncogene.

The article "MiRNA-211 suppresses cell proliferation, migration and invasion by targeting SPARC in human hepatocellular carcinoma" was retracted in 2023. Reasons: duplicated images; duplicated data; original data or images not available.

### Suppression of SPARC was functionally important for the biological effects of miR-211

To explore the functional significance of SPARC in the proliferation and invasive capability of HCC cells induced by miR-211, we ectopically expressed open reading frames of SPARC to assess whether these ORFs may rescue the suppression effect induced by miR-211. Interestingly, the growth inhibitory phenotypes were partly alleviated by SPARC re-expression in 97H-miR-211 and LM3-miR-211 cells (MTT proliferation assay, Fig. 6A). The motility-inhibitory effects of miR-211 were also partially abrogated by SPARC re-expression (wound healing assay, Fig. 6B; Matrigel-coated transwell assay, Fig. 6C). Previous studies have shown that SPARC suppressed the mobility of melanoma cells by repressing expression of E-cadherin^25^. Then we detected the expression of metastasis-associated proteins. Expressions of SPARC, vimentin, N-cadherin, MMP-2 and MMP-9 were decreased but E-cadherin was uniformly showed up-regulated in miR-211 ectopic expression cells. Moreover, reintroduction of SPARC reversed the miR-211 inhibition of metastasis-associated proteins (Fig. 6D). These results demonstrated that SPARC was functionally important in the role of miR-211 in cell proliferation, migration and invasion in HCC.

## Discussion

Previous studies have suggested that miR-211 inhibits cell proliferation and invasion in many different cancers^13^,^14^,^15^. However, the expression and function of miR-211 in HCC as well as the molecular mechanisms by which miR-211 exerts its functions and regulates the phenotypic diversity of HCC cells have not been fully understood. Our present study suggests the first comprehensive analysis of miR-211 in hepatocellular carcinoma. MiR-211 was downregulated in HCC tissue and reduced miR-211 levels were significantly correlated with HCC progression and poor patient survival, suggesting that miR-211 might play an important role as a suppressor of growth and metastasis in HCC progression and represent a potential target for HCC therapy.

In this study, the expression level of miR-211 was detected in HCC cells and tissues by real-time quantitative PCR. We found that miR-211 expression was significantly lower in human HCC tissues than that of adjacent normal tissues, consistent with previous report^13^. Moreover, our analysis results showed that the expression level of miR-211 was significantly correlated with tumor vein invasion, TNM stage and overall HCC survival. These results suggest that miR-211 might play a role in HCC tumoregenisis as a potential tumor suppressor.

The article "MiRNA-211 suppresses cell proliferation, migration and invasion by targeting SPARC in human hepatocellular carcinoma" was retracted in 2023. Reasons: duplicated images; duplicated data; original data or images not available.

Then the putative tumor suppressor function of miR-211 was assessed in human HCC by *in vitro* and *in vivo* assays. Ectopic expression of miR-211 in the 97H and LM3 significantly inhibited cell proliferation as evidenced by cell viability and colony formation assays. Furthermore, we performed FACS to evaluate the effects of miR-211 on apoptosis levels and found that overexpression of miR-211 increased apoptosis. In addition, the ectopic expression of miR-211 displayed a significantly lower growth rate than the control cancer cells *in vivo*. Tumor metastasis is the leading causes of cancer mortalities and involves in a series of genes related to biological progression in various tumors^1^,^29^, it would be interesting to investigate whether miR-211 contributes to cell migration and invasion. Our results indicated that overexpression of miR-211 notably inhibited cell migration and invasion. In accordance with our *in vitro* findings, ectopic expression of miR-211 led to fewer metastatic loci compared with vector control cells, providing *in vivo* evidence that miR-211 has therapeutic potential for metastasis prevention. On the other hand, however, some studies have shown that miR-211 promoted colorectal cancer cell growth *in vitro* and *in vivo* and acted as a tumor-promoting miRNA^18^. This discrepancy may be attributed to a tissue specific function of miR-211 in HCC compared with other tumors. Our results suggest that miR-211 may function as a negative regulator or tumor suppressor for cell proliferation, invasion and metastasis in HCC.

The molecular mechanisms involved in miR-211-mediated repression of growth and metastasis are not well understood. SPARC was sought for the possible gene effectors participating in miR-211 function. We confirmed the SPARC 3′UTR as a direct target of miR-211 by dual-luciferase assays and western blotting. Elevated SPARC expression was also related with tumor invasion and metastasis in several solid cancers, such as melanoma^23^, HCC^27^, gliomas^20^, and gastric cancer^22^. In the present study, we found that SPARC expression was significantly increased in HCC samples compared with paired adjacent normal tissues. Knockdown of SPARC could phenocopy the effects of miR-211 overexpression. Additionally, further study indicated that the expression of SPARC could partially restore the inhibition functions of miR-211. Meanwhile, it has been reported that SPARC modulates the protein level of E-Cadherin, which mediated cell-cell adhesion played a critical role in development of invasive tumors^25^,^30^. In the current study, we found that overexpression of miR-211 could suppress the expression of SPARC, followed by downregulation of metastasis-associated proteins.

The article "MiRNA-211 suppresses cell proliferation, migration and invasion by targeting SPARC in human hepatocellular carcinoma" was retracted in 2023. Reasons: duplicated images; duplicated data; original data or images not available.

## Conclusions

In summary, we have identified that miR-211 was frequently downregulated in HCC, which was correlated with HCC progression and survival. MiR-211 overexpression inhibits cell growth and metastasis both *in vitro* and *in vivo* by directly targeting SPARC. The involvement of miR-211 mediated SPARC downregulation may yield further insight into the molecular mechanisms underlying cancer aggressiveness.

## Materials and Methods

### Patients and clinical samples

Investigation has been conducted in accordance with the ethical standards and according to the Declaration of Helsinki and according to national and international guidelines and has been approved by the Ethics Committee of Shanghai First People’s Hospital. Written informed consent was obtained from each patient who participated in the investigation. Matched fresh frozen primary tumor samples and corresponding non-tumorous tissue used in this study were obtained from 227 patients who underwent HCC resection at the Department of General Surgery, Shanghai First People’s Hospital of Shanghai Jiao Tong University from May 2006 to July 2009. All patients were positive for hepatitis B virus (HBV) infection. Follow-up data were obtained after hepatic resection to assess survival rates and to monitor recurrence and metastases. The relevant clinical characteristics of the HCC patients are shown in Table 1.

### Cell lines and cell culture

Human HCC cell lines (MHCC-LM3, MHCC-97H, MHCC-97L, SMMC-7721, and HepG2), the normal human hepatic cell line LO2, and human embryonic kidney cell lines (HEK293T)were grown in Dulbecco’s modified Eagle’s medium (Thermo Scientific Hyclone, Rockford, IL, USA) that was supplemented with 10% fetal bovine serum (Life Technologies, Inc. Rockville, MD, USA) and 1% penicillin/streptomycin (Life Technologies) in a humidified atmosphere of 5% CO_2_ at 37 °C.

### Plasmids, lentivirus production and transduction

DNA fragments containing the hsa-miR-211 precursor with at least 250 bp flanking sequence of each side were amplified from human genomic DNA and inserted into the BamHI and MluI sites of the pWPI.1 vector. The coding sequences of SPARC was amplified and cloned into pcDNA3.1 (+) to generate SPARC expression vectors. The wild-type 3′-UTR segment of human SPARC containing the predicted target sites of miR-211 were kindly provided by Dr Zhu (Fudan University, Shanghai, China). The mutant 3′-UTR of SPARC, which have the mutated sequences (“CAAAGGGAA” as “CACCGCCGA”) in the complementary sites of the seed region of miR-211, were generated by site-specific mutagenesis based on psi- SPARC-3′ UTR-WT. All constructs were verified by sequencing.

The article "MiRNA-211 suppresses cell proliferation, migration and invasion by targeting SPARC in human hepatocellular carcinoma" was retracted in 2023. Reasons: duplicated images; duplicated data; original data or images not available.

Lentivirus particles were harvested 60 h after either an empty pWPI.1 vector or pWPI-miR-211 was transfected into HEK-293T cells using Lipofectamine 2000 reagent (Invitrogen) with the packaging plasmid psPAX2 or pMD2.G. Target cells were grown to 40% confluence and infected with recombinant lentivirus-transducing units plus 8 mg/ml Polybrene (Sigma, St Louis, MO, USA).

### RNA extraction and quantitative real-time PCR

Total RNA was extracted from cultured cells and from surgically resected fresh HCC tissues using Trizol Reagent (Life Technologies) according to the manufacturer’s instructions. Then, 5 ng of total RNA was reverse transcribed using a TaqMan miRNA Reverse Transcription Kit (Applied Biosystems, Foster City, CA, USA), and the expression levels of mature forms of miR-211 was determined using an miRNA-specific TaqMan MiRNA Assay Kit. Relative fold changes of expression were normalized to U6 expression. To determine the mRNA levels of SPARC, total RNA (500 ng) was reverse transcribed using PrimeScript® RT Master Mix (TaKaRa, Dalian, China) reverse transcriptase according to the manufacturer’s instructions, and qRT-PCR analyses were performed using FastStart Universal SYBR Green Master (Roche, Mannheim, Germany). Data were normalized to GAPDH expression. All analyses were performed using the ABI PRISM® 7900HT Sequence Detection System, and the comparative delta CT method was used to calculate relative expression. Primers were as follows: SPARC forward, 5′ AGCACCCCATTGACGGGTA 3′, reverse, 5′ GGTCACAGGTCTCGAAAAAGC 3′; GAPDH forward, 5′ CTGGGCTACACTGAGCACC3′, reverse, 5′ AAGTGGTCGTTGAGGGCAATG 3′.

### Luciferase reporter assays and siRNA transfection

HEK293T cells were cultured in 96-well plates and transiently co-transfected with wild-type or mutated reporter plasmid and pWPI.1 vector or pWPI-miR-211 vector. For the antagonism experiment, 97H, stable overexpression miR-211, were transiently transfected with wild-type or mutant reporter plasmid and inhibitor NC (anti-miR-control) or anti-miR-211 (miR-211 inhibitors). All synthetic Negative Control anti-miR inhibitor and anti-miR-211 were purchased from Applied Biosystems. Dual luciferase reporter assays (Promega) were analyzed 48 h after transfection. Transfections were performed in triplicate and repeated in at least three independent experiments.

The article "MiRNA-211 suppresses cell proliferation, migration and invasion by targeting SPARC in human hepatocellular carcinoma" was retracted in 2023. Reasons: duplicated images; duplicated data; original data or images not available.

To silence SPARC expression, target cells were transfected with SPARC-specific siRNA or a negative control. siRNA against SPARC significantly reduced the expression of SPARC in comparison with control siRNA in transfected cells in protein levels.

### Cell proliferation and colony formation assay

Cell proliferation assays were conducted using cell counting kit-8 (CCK-8) (Dojindo Laboratories, Kumamoto, Japan) according to the manufacturer’s instructions. A total of 3 × 10^3^ cells were seeded into a 96-well plate and cultured in 100 μL normal culture medium. CCK-8 reagent was added at the indicated time points after seeding and incubated at 37 °C for 2 h. Absorbance was measured for each well at 450 nm using a microplate reader (TECAN, Switzerland). Each experiment was performed in triplicate and repeated at least 3 times independently.

For colony formation assays, 500 cells per well were plated in 6-well plate (Corning) with 10% FBS for 14 days. Cells were fixed for 15 minutes and stained with 1% crystal violet for 30 minutes. Colonies with more than 50 cells per colony were counted. All of the experiments were performed in triplicate repeated at least 3 times independently.

### Cell invasion assay and wound healing assay

For the cell invasion assay, a filter membrane with an 8-μm pore size (Corning, NY, USA) was coated with 25 μl of Matrigel (BD Biosciences, Bedford, MA, USA) and 75 μl of culture medium without FBS. Then, 100 μl of the cell suspension (3 × 10^4^ cells) was added to the Transwells with 600 μl of complete medium in the lower chamber. After incubation for 48 h, the cells that invaded through the Matrigel membrane were fixed and stained with 1% crystal violet for 30 minutes. 6 random microscopic fields of each insert were counted using an Olympus light microscope.

A total of 1 × 10^4^ cells were seeded into a 24-well plate for 24 h. Cells were disrupted by scraping with a 200 μl pipette tip and then washing with medium to remove the displaced cells. The scrape width was measured under the Olympus light microscope and analyzed by NIH Image J software at 24 h later.

### Apoptosis assay

After incubation at 37 °C in 5% CO_2_, the cells were harvested and washed twice with cold PBS. Cells were resuspended and stained with Annexin V-PE and propidium iodide (PI) using the Annexin V-PE Apoptosis Detection Kit I (BD Biosciences) for 20 min at room temperate in the dark. Then cells were analyzed using a Flow Cytometer (BD Biosciences, San Jose, CA) according to manufacturer’s instructions. All experiments were performed in triplicate.

### *In vivo* tumorigenicity and tail vein metastasis analysis

This experiment was approved by Experimental Animal Ethics Committee of Shanghai Jiao Tong University with the permit number of 20130421-GR. All procedures were carried out in accordance with the NIH Guide for the Care and Use of Laboratory Animals and local institutional ethical guidelines for animal experiment. 5 × 10^6^ LM3 cells (suspended in 0.1 ml sterile PBS) infected with either pWPI.1 vector or pWPI-miR-211 vector as described above were injected subcutaneously in the front legs of the 4-week-old BALB/c-nu/nu male mice (6 per group, Slaccas, Shanghai). Tumor volumes were monitored by measuring the length (L) and width (W) of the tumor once a week using a digital caliper and were calculated with the following formula: tumor volume (mm3) = L × W^2^ × 0.5. Mice injected with LM3-vector or LM3-miR-211 cells were sacrificed 7 weeks after injection. To study lung metastasis, 1 × 10^6^ cells (LM3-vector or LM3-miR-211) in 200 μl PBS were injected into the tail vein of 6-week-old BALB/c nude mice (6 per group), which were injected intraperitoneally with a 2 mg/kg dose of LPS. Mice were sacrificed 5 weeks after the injections. The lungs of each mouse were excised, and serial sections of the lungs were stained with H&E; then the number of metastatic foci, was counted under a light microscope.

The article "MiRNA-211 suppresses cell proliferation, migration and invasion by targeting SPARC in human hepatocellular carcinoma" was retracted in 2023. Reasons: duplicated images; duplicated data; original data or images not available.

### Immunohistochemistry

Paraffin embedded tissue microarray (TMA) slides consisted of 227 HCC samples. Sections were deparaffinized and re-hydrated according to standard protocols, and heat-induced antigen retrieval was performed in 0.01 M sodium citrate buffer (pH 6.0). Endogenous peroxidase activity was quenched by 3% hydrogen peroxide, and the slides were washed with TBS and blocked with goat serum for 15 minutes. Then, they were incubated with primary antibody against SPARC (Cell Signaling, Danvers, MA, USA) overnight at 4 °C. Non-immune IgG was used as a negative control. The reaction products were visualized with the EnVision system (DAKO). The expression of SPARC was assessed by two pathologists who were blinded to the experimental protocol. The proportion score was according to the percentage of SPARC -positive cells (0, none; 1, < = 10%; 2, 10 to < = 25%; 3, > 25 to 50%; 4, >50%). For statistics, the general intensity score value was calculated by multiplying the intensity score by the extent score, for a range from 0 to 11. The SPARC expression was determined as negative (score 0–1), weak (score 2–5), moderate (score 6–8), or strong (score 9–11).

### Immunoblotting

Protein was extracted from the cancer cell lines and tumor tissues and was lysed with RIPA lysis buffer (Cell Signaling) with proteinase inhibitor. Equal amounts of protein were separated by 10% SDS- polyacrylamide gel electrophoresis and transferred to PVDF membranes (Bod-Rad, Hercules, CA, USA), which were blocked with 1% BSA in Tris-buffered saline containing 0.1% Tween-20. The membranes were incubated overnight at 4 °C with primary antibodies (Anti-E-cadherin, Anti-N-cadherin and Anti-Vimentin from Cell Signaling; Anti-MMP2 and Anti-MMP-9 from Abcam), with GAPDH (Cell Signaling) as the loading control. After incubation, the membranes were incubated with the appropriate HRP-conjugated secondary antibody for 1 hour at room temperature. Protein bands were detected with chemiluminescent substrate detection (Thermo Fisher Scientific Inc., Waltham, MA, USA) visualized on Laser4000 (Fujitsu, Stamford, CT). The bands were subjected to quantification using the ImageJ imaging processing program (National Institutes of Health).

The article "MiRNA-211 suppresses cell proliferation, migration and invasion by targeting SPARC in human hepatocellular carcinoma" was retracted in 2023. Reasons: duplicated images; duplicated data; original data or images not available.

### Statistical analysis

Data is expressed as mean ± SD of triplicate experiments. Statistical analysis was performed using Student’s t test. Survival curves were assayed using the Kaplan-Meier method. Pearson χ2 test was used for analyzing the correlations between the expression level of miR-211 and clinicopathologic features of patients. P value < 0.05 was considered statistically significant for all tests.

## Additional Information

**How to cite this article**: Deng, B. *et al.* MiRNA-211 suppresses cell proliferation, migration and invasion by targeting SPARC in human hepatocellular carcinoma. *Sci. Rep.* **6**, 26679; doi: 10.1038/srep26679 (2016).

## Figures and Tables

**Figure 1:** Down-regulation of miR-211 in HCC correlated with worse clinical outcomes. (**A**) miR-211 expression in indicated human HCC cell lines and immortalized human hepatic cell line (L02). (**B**) Relative expression of miR-211 in 227 pairs of HCC tissues (Tumor) and their corresponding adjacent non-cancerous tissues (Non Tumor). Expression levels of miR-211 were normalized to U6 expression. (**C**) Kaplan-Meier curve of correlation between the miR-211 level and overall survival of 2 groups of high (greater than the mean; n = 117) and low (less than the mean; n = 110) miR-211 expression levels in the primary tumors from 227 HCC patients. (**D,E**) Kaplan-Meier analysis of the survival of HCC patients according to their UICC stage: UICC I-II subgroup, UICC III-IV subgroup. **P < 0.01.

**Figure 2:** Overexpression of miR-211 inhibits cell proliferation *in vitro*. (**A**) Real-time RT-PCR analysis of the expression levels of miR-211 in 97H and LM3 cells stably expressing miR-211. (**B**) Cell proliferation rate of 97H and LM3 cells transfected with vector or miR-211by MTT assay. (**C**) Representative photographs (left) and relative quantification (right) of colony formation were counted in an anchorage-independent growth ability assay. (**D**) Cell apoptosis was assessed by flow cytometric analysis in 97H and LM3 cells. (**E**) Overexpression of miR-211 inhibited tumor growth *in vivo*. Representative tumor xenografts excised from nude mice administered a subcutaneous injection of LM3-vector or LM3-miR-211 (left). Quantification of tumor mass weight (right). Data are presented as the mean ± SD. (**F**) Representative immunohistochemical staining of Ki67 in tumor xenografts excised from nude mice. **P < 0.01.

The article "MiRNA-211 suppresses cell proliferation, migration and invasion by targeting SPARC in human hepatocellular carcinoma" was retracted in 2023. Reasons: duplicated images; duplicated data; original data or images not available.

**Figure 3:** miR-211 suppressed tumor migration and invasion *in vitro* and *in vivo*. (**A**) Representative micrographs of wound length at 0 and 24 h after wounding. The indicated cells transfected with either vector or miR-211 (left) and a histogram showed the rate of front migration of cells of 5 randomly selected fields. (**B**) Representative photographs of Matrigel invasion assays at 36 hours after seeding. The indicated cells transfected with either vector or miR-211 (left) and quantification of indicated invading cells in 5 random fields. (**C**) Representative images of lung metastases in nude mice by tail vein injection were confirmed by H&E staining. Data are presented as the mean ± SD based on three independent experiments. **P < 0.01.

**Figure 4:** miR-211 regulation of SPARC expression. (**A**) Computational algorithm showed that the putative miR-211-binding sequence was in the 3′UTR of SPARC. (**B**) Luciferase reporter construct containing wild-type or mutated SPARC 3′UTRs were cotransfected with vector or miR-211 into 293T cells. (**C**) 97H cells that were stably overexpressing miR-211 were transfected with either the wild-type or mutated SPARC 3′UTR, along with control inhibitors (inhibitor-NC) or miR-211 inhibitor (Anti-miR-211). Relative Renilla luciferase activity was measured at 48 hours after transfection and normalized to firefly luciferase. (**D**) The mRNA expression of SPARC in 97H and LM3 cells stably expressing miR-211. (**E**) The endogenous expression of SPARC was determined by western blotting analysis in 97H and LM3 cells transfected with vector or miR-211. (**F**) The endogenous protein expression of SPARC in 97H and LM3 cells stably overexpressing miR-211 and transfected with inhibitor-NC or miR-211 inhibitor was analyzed by western blotting. **P < 0.01.

**Figure 5:** SPARC was significantly upregulated in HCC tissues, and its expression was inversely correlated with miR-211 expression. (**A**) The mRNA expression of SPARC in 227 pairs of HCC tissues (Tumor) and their corresponding adjacent non-cancerous tissues (Non Tumor). (**B**) A statistically significant inverse correlation between miR-211 and SPARC mRNA levels in the 227 cases of HCC tissues. U6 and GAPDH were used as an internal control. (**C**) Representative images of low SPARC and high SPARC immunohistochemical staining in human HCC samples. Magnification: x100. (**D**) Spearman’s correlation analysis of SPARC IHC and the expression level of miR-211. Corresponding P values analyzed by t-test or Spearman correlation test were as indicated. (**E**) Western blot analysis of SPARC in 97H and LM3 cells transfected with scramble sequence (SCR) or siSPARC. (**F**) Apoptosis analysis of 97H and LM3 cells transfected with scramble sequence (SCR) or siSPARC. (**G**) Wound healing assay and invasion assay (**H**) were analyzed in 97H and LM3 cells transfected with scramble sequence (SCR) or siSPARC. **P < 0.01.

The article "MiRNA-211 suppresses cell proliferation, migration and invasion by targeting SPARC in human hepatocellular carcinoma" was retracted in 2023. Reasons: duplicated images; duplicated data; original data or images not available.

**Figure 6:** SPARC was functionally involved in the miR-211-mediated proliferation and invasion of HCC cells. (**A**) MTT assay, (**B**) Wound healing assay and (**C**) invasion assay were analyzed in 97H-miR-211 and LM3-miR-211 cells transfected with control (control) or SPARC. (**D**) Total lysates from the indicated cells with different treatments were analyzed with relative antibodies by WB analysis. GAPDH was used as the loading control.

**Table 1:** Associations between miR-211 expression levels and clinicopathologic features of HCC patients.

Clinicopathologic Variables	n	Low	High	P
		(n = 117)	(n = 110)	
Sex				
Female	29	12(5%)	17(7%)	0.320
Male	198	105(46%)	93(41%)	
Age, y				
≤50	99	53(23%)	46(20%)	0.688
>50	128	64(28%)	64(28%)	
Preoperative AFP(ng/mL)				
≤20	88	46(20%)	42(19%)	0.892
>20	139	71(35%)	68(30%)	
Liver cirrhosis				
No	71	32(14%)	39(17%)	0.200
Yes	156	85(37%)	71(32%)	
ALT(units/L)				
≤75	158	74(32%)	84(37%)	0.274
>75	69	33(15%)	36(16%)	
Tumor size(cm)				
≤5	143	81(36%)	62(27%)	0.168
>5	84	39(17%)	45(20%)	
Tumor number				
Single	144	78(34%)	66(29%)	0.335
Multiple	83	39(17%)	44(20%)	
Vein invasion				
No	180	94(41%)	86(38%)	**0.0028**
Yes	47	36(16%)	11(5%)	
TNM stage				
I–II	138	58(25%)	80(36%)	**0.0004**
III–IV	89	59(26%)	30(13%)	

All analyses were conducted on 227 cases using χ^2^ tests. Median value of all 227 cases was chosen as the cut-off point for distinguishing miR-211 low-expression tumors from miR-211 high-expression cases.
